# Integrated Analysis of Multiomics Data Identified Molecular Subtypes and Oxidative Stress-Related Prognostic Biomarkers in Glioblastoma Multiforme

**DOI:** 10.1155/2022/9993319

**Published:** 2022-09-22

**Authors:** Yawen Ma, Zhuo Xi

**Affiliations:** Department of Neurosurgery, Shengjing Hospital of China Medical University, Shenyang, Liaoning 11000, China

## Abstract

Glioblastoma multiforme (GBM) is a glioma in IV stage, which is one of the most common primary malignant brain tumors in adults. GBM has the characters of high invasiveness, high recurrence rate, and low survival rate and with a poor prognosis. GBM implicates various genetic changes and epigenetic and gene transcription disorders, which are crucial in developing GBM. With the progression and enhancement of high-throughput sequencing technologies, the acquirement and administering approaches of diverse biological omics data on distinctive levels are developing more advanced. However, the research of GBM with multiomics remains largely unknown. We identified GBM-related molecular subtypes by integrated multiomics data and exploring the connections of gene copy number variation (CNV) and methylation gene (MET) change data. The expression of CNV and MET genes was examined through cluster integration analysis. The present study confirmed three clusters (iC1, iC2, and iC3) with distinctive prognosis and molecule peculiarities. We also recognized three oxidative stress protecting molecules (OSMR, IGFBP6, and MYBPH) by contrasting gene expression, MET, and CNV in the three subtypes. OSMR, IGFBP6, and MYBPH were differentially expressed in the clusters, suggesting they might be recognized as characteristic markers for the three clusters in GBM. Through integrative investigation of genomics, epigenomics, and transcriptomics, we offer novel visions into the multilayered molecules of GBM and facilitate the accuracy remedy for GBM sufferers.

## 1. Introduction

Glioblastoma multiforme (GBM) is one of the central nervous system's most common and highly malignant primary tumors [1]. The incidence rate of GBM in men is higher than that in women, with a tendency for family aggregation [2]. Previous studies suggest that the average onset of GBM is about 60 years old; however, the patients showed a younger trend in recent years. The common symptoms of GBM are progressive somatosensory and motor dysfunction, headache, dizziness, and convulsions [3, 4]. At present, surgical resection is the standard method for treating GBM. Postoperative temozolomide concurrent radiotherapy and chemotherapy followed by temozolomide oral chemotherapy were the primary treatment for GBM. However, even after active treatment, the prognosis of GBM is still inferior [5]. In recent years, the development of high-throughput technology and bioinformatics analysis has dramatically increased the amount of biological data for research and provided new ideas for exploring the etiology, pathogenesis, and new drug treatment targets of GBM [6, 7].

High throughput technology is applied to various “omics,” mainly including (1) genomics, which is used to detect DNA mutations; (2) transcriptomics, which is used to detect mRNA expression; (3) epigenomics which studies the effect of DNA modification on mRNA expression without changing the sequence; (4) proteomics, which is used to detect protein components; and (5) metabonomics, used to determine the level of metabolites [8]. Omics technology could evaluate and integrate omics data of tissues and cells, accurately exhibit the biological process of disease, and facilitate the realization of personalized precision medicine [9]. Genomic change resulting from gene CNV and single-nucleotide mutations (SNPs) might accelerate the progression of cancers [10]. CNV plays a crucial supervisory role in GBM development, and transcriptional dysregulation resulting from copy number alterations was future actions in GBM development [11]. In addition, exploration of DNA MET has validated the massive heterogeneousness of epigenome obstacles in GBM and various cancers. Emerging evidence shows that DNA methylation facilitates heterogeneous biologic activities and is implicated in GBM development. The multiomics profiles enable it feasible to carry out an integrated exploration based on genomics, epigenomics, and transcriptomics to enhance GBM prognosis [12].

In this study, we evaluated gene expressions using genomic and epigenetic patterns using a multi-omics combination. We also determined distinctive molecular subtypes markedly related to GBM outcome. Three oxidative stress-related prognostic biomarkers for patients with GBM were identified based on CNV, MET, and gene expressions.

## 2. Methods

### 2.1. Data Origination

R software was employed to analyze the clinical data, RNA-seq, methylation, and CNV from The Cancer Genome Atlas (TCGA) GBM cohorts. At the same time, SNV data from TCGA GBM is also obtained. We next sought datasets about the GBM miRNA expressions from the Gene Expression Omnibus (GEO) database. The microarray dataset GSE4271, including GBM clinical patients, was selected for our subsequent analysis.

### 2.2. Data Processing

About the arrangement of CNV probes, two intervals with 50% overlap were regarded as equivalent, whereas the number of coverages probes less than five intervals was uninvolved. They were mapping CNV probes to corresponding genes using GTF of GENCODE. The GRh38's Gencode.v22 was used for CNV intervals mapping to the related gene. About RNA-seq statistics, the low expression genes in each trial were uninvolved (the proportion of samples with 0 per kilobase of transcript per million mapped reads (FPKM) per million mapping reads to the total sample was <0.5), whereas the gene set with advanced expression was reserved. About chip statistics, directly load the standardized expression profile (EXP) matrix and reach the probe with the gene consistent with the note of the platform. The median level of multiple probes matched to a similar gene was established as the gene expression, whereas probes matched to compound genes were detached. For the methylation data, exceeding 70% of the trials existed omitted spots, which were replaced with values created through the KNN (*k*-Nearest Neighbor) approach. Using GRh38's Gencode.v22 comment preserved TSS probes of 200 bp downstream and 2 kb upstream and further recorded their genes.

### 2.3. Detection of CNV-G and MET-G Gene Set

This study used the Pearson correlation coefficient (*R*) to evaluate the correlation among RNA-seq, DNA methylation, and CNV. The correlation coefficient is transformed to a *Z* value conferring to ln ((1 + *r*)/(1 − *r*)). The genes that scored *P* < 0.05 in the correlation coefficient assessment established a gene set drastically associated with (CNV genes) CNV-Gs and another gene set associated with MET-Gs (methylation genes).

### 2.4. The Molecular Subtype Identification

The iClusterPlus package and nonnegative matrix factorization (NMF) in R software were used to discover the genomics-based molecular subtypes between the expressions of CNV-G/MET-G gene sets. To observe the association between the CNV-G/MET-G gene sets and phenotypes, the trials were clustered by the NMF technique. The clinical characteristics of the samples and the connection between the molecular subtypes were studied. Cluster K was established as 2-10. According to the correlation coefficient, the ideal clusters of molecular subgroups were established based on CNV-Gs and molecular subgroups based on MET-Gs.

### 2.5. Association between Molecular Subtypes and Tumor Microenvironment

TIMER is an approach used to systematically evaluate the clinical effect of diverse immune cells on different tumors. The CIBERSORT method was applied to assess the distribution of immune cells in all tumor trials, and when the samples with *P* < 0.05 were elected for correlation analysis between immune cells and target genes.

### 2.6. Exploration of Genetic Alterations in Molecular Subtypes

Genetic differences in distinctive molecular subtypes were assessed. DESeq2 was applied to explore variances in gene expressions between diverse molecular subtypes, and two-fold difference criteria plus FDR < 0.05 was chosen as the threshold to distinguish genetic differences across molecular subtypes.

### 2.7. Association between Genomic Variation and Molecular Subtypes

To uncover the association between genomic deviation and molecular subtypes, TCGA-GBM statistics were examined. Fisher's exact test was applied to examine the differentially expressed genomic. *P* < 0.05 was chosen to detect mutational variances.

### 2.8. Statistical Analysis

Spss20.0 statistical analysis software was used for data analysis, and the Pearson linear correlation test was applied to examine the correlation. Log-rank and Kaplan–Meier (KM) tests were used for survival analysis. *P* < 0.05 was considered statistically significant.

## 3. Results

### 3.1. Comparison of CNV-Gs and MET-Gs

664 CNV-Gs and 1316 MET-Gs were identified using correlation analysis with *P* < 0.05. As shown in Figure 1(a), the correlation of CNV-Gs markedly transferred to the right, whereas the correlation of MET-Gs transferred to the left. Furthermore, the association between CNV and gene expressions was evaluated, and we observed the overall correlation coefficient > 0, implying that CNV was positively connected to gene expressions (Figure 1(a)). A comparison of CNV-Gs and MET-Gs gene sets observed 50 overlapping genes (Figure 1(b)). We found a notable difference in the distribution of CNV-Gs on chromosomes 1 and 2 (Figure 1(c)). Similarly, we also observed a marked difference in the MET-G distribution on chromosomes 1 and 2 (Figure 1(d)). We observed marked differences in the frequency of DNA methylation in vivo and at the transcription initiation site (Figure 1(e)). In addition, most MET-Gs were observed in the open sea regions than in CpG islands (*P* < 0.001, Figure 1(f)).

### 3.2. CNV-G and MET-G Gene Set-Based Molecular Subtype Detection

To distinguish molecular subtypes that exposed the multiomics forms of the CNV-G and MET-G gene sets, the genomic statistics of CNV, MET, and RNA expressions were integrated through the iCluster. Three clusters (iC1, iC2, and iC3) were identified for CNV-Gs by the NMF method (Figure 2(a)). Similarly, three ideal clusters (iC1, iC2, and iC3) were obtained for MET-Gs (Figure 2(b)). As shown in Figure 2(c), marked prognostic changes were detected in the three CNV-G subtypes. Moreover, the three MET-G subtypes detected marked prognostic differences (Figure 2(d)). Most importantly, we found an apparent overlap among the three CNV-G subtypes and three MET-G subtypes (Figure 2(e)).

### 3.3. MET, CNV, and EXP Data Were Integrated into Cluster Samples

By clustering the omics data, we obtained three subtypes (iC1, iC2, and iC3) with noticeably altered OS times. A heatmap was screened to exhibit the RNA gene expression of CNV-G and MET-G clusters (Figure 3(a)). Moreover, it is determined that the OS time of the three subtypes (iC1, iC2, and iC3) was considerably different, and iC3 had the worst OS among the three clusters (Figure 3(b)).  Figure 3(c) shows iC2 had a markedly better OS than iC1. Furthermore, iC1 had a markedly better OS than iC3 (Figure 3(d)). iC2 had a markedly better OS than iC3 (Figure 3(e)). These results implied that iC2 had the best OS time in the three subtypes.

### 3.4. DNA CNV Abnormalities Were Accordant with MET Abnormalities

To assess the association between CNV and methylation aberrations, CNV > 0.3 was considered gain, CNV < −0.3 was considered loss, the *β* value of MET > 0.8 was classified as MetHypo, and MET < 0.2 was classified as MetHypo. As shown in Figure 4(a), a marked correlation existed between CNV loss and gain. However, the correlation between Gain and MetHype/MetHypo, loss, and MetHyper/MetHypo was not statistically different (Figures 4(b)–4(e)). In addition, MetHypo is negatively connected to methyper (Figure 4(f)).

### 3.5. Analysis of Tumor Immune Cell Infiltration in Molecular Subtypes

The CIBERSORT algorithm was applied to compare tumor immune cell infiltration in subtypes and determine the proportions of the tumor-infiltrating immune cells in distinctive subtypes (Figure 5(a)). The percentage of tumor immune cell infiltration in tissue samples from patients with GBM was determined (Figure 5(b)). Most importantly, we observed an increased percentage of neutrophils in the iC2 subtype compared to other subtypes (Figure 5(c)).

### 3.6. Molecular Characteristics of the Three GBM Subtypes

According to the findings of iCluster, gene expression changes between the three subtypes with prognostic distinctions were compared, and 564 DEGs were identified, followed by the removal of low-expressed genes (Figure 6(a)). The methylation incidence of DEGs in iC2 was markedly enhanced compared with that of iC1 and iC3, implying that methylation exhibited specific impacts on GBM prognosis (Figure 6(b)). When assessing the relationship between gene expression, MET, and CNV, we observed that the gene expression of DEGs in trials with MET was markedly enhanced (Figure 6(c)). The GO enrichment evaluation showed that the DEGs were markedly enriched in an extracellular matrix organization, angiogenesis cell differential, and regulation of nervous development (Figure 6(d)). Similarly, the enriched KEGG pathways of the DEGs are demonstrated in Figure 6(e).

### 3.7. Association between Gene Expressions and CNV/MET

To explore the association between gene expressions and CNV-Gs/MET-Gs, the survival analysis was performed to recognize the differentially expressed genes among three subtypes. Three genes, OSMR, MYBPH, and IGFBP6, were markedly connected to prognosis. The expression of MYBPH and the IGFBP6 gene were negatively correlated with MET (Figures 7(b) and 7(d)). However, there was no difference between the expression of MYBPH and IGFBP6 genes and CNV (Figures 7(a) and 7(c)). MYBPH and IGFBP6 were markedly advanced in iC2 with the wickedest prognosis than iC1 and iC3 (Figures 7(e) and 7(f)). In addition, we uncovered that the expression of MYBPH and IGFBP6 expression was appreciably connected to tumor prognosis (Figures 7(g) and 7(h)).

### 3.8. Mutation Spectrum of the Three GMB Subtypes

We studied whether the mutation spectrum of the three GBM subtypes is different. To detect the top 50 genes, the mutation spectrum of different subtypes was evaluated (Figures 8(a) and 8(b)). Through evaluating the mutation spectrum variances, we uncovered that the gain/loss of CNV in iC2 was much more marked higher than in iC1 and iC3 subtypes (Figure 8(c)). By comparing the iC2 subtype with the other two subtypes, we found that TP53, PTEN, NF1, EGFR, AHNAK TTN, MUC16, and AHNAK2 were the top eight common mutant genes (Figures 8(d) and 8(e)).

## 4. Discussion

Glioblastoma multiforme (GBM) belongs to grade IV glioma and accounts for 12% to 15% of all intracranial tumors. It has the highest malignant degree and the worst prognosis in gliomas, and the 5-year survival rate is only 5% [13]. Similar to other malignant tumors, glioblastoma has the characteristics of high invasion, resistance to radiotherapy and chemotherapy, immunosuppression in the microenvironment, and a high recurrence rate [14]. Operation combined with radiotherapy and chemotherapy is the standard treatment for GBM [15]. However, despite the increasing understanding of glioblastoma, there is still a lack of practical progress in treating this disease. Therefore, there is an urgent need to make new progress in studying the exact molecular mechanisms and reliable therapeutic targets of GBM.

Emerging evidence indicates that cancer results from abnormal genetic and epigenetic events [16]. The epigenetic mechanism is a stable genetic feature that changes in DNA sequence could not explain [17]. Like histone modification, DNA methylation does not affect the genome DNA sequence but adds a methyl (CH3) group to CG dinucleotide cytosine [18]. According to the abnormal changes in DNA methylation, diagnosing and treating tumors and predicting biomarkers are considered broad prospects [19]. In recent years, most of the studies have focused on the kinetics of aberrant promoter methylation in GBM, and there are also a few studies on enhancer methylation. Aberrant methylation enhancers can lead to various diseases, including abnormal gene expression in various cancers [20, 21].

An in-depth understanding of genetic and epigenetic variations might assist in elucidating the pathogenesis of GBM. In the current study, we used multiomics data from TCGA GBM and GSE4271 datasets to identify the molecular subtypes and oxidative stress-related prognostic biomarkers in glioblastoma multiforme. We evaluated the association between epigenetics and CNV and detected that DNA CNV deviations were constant with MET aberrations. Through multiomics relationship investigation, CNV-C and MET-C gene sets were recognized, and the association between CNV and MET was created with the gene expressions. According to multiomics clusters constructed with gene expression, MET, and CNV, three molecular subtypes were obtained; iC2 was related to the poorest clinical results. Additionally, we recognized three prognostic gene indicators and validated them as well.

The immunophenotype of the tumor microenvironment functions a critical role in tumor occurrence and progress and is crucial for the prognosis and success of immunotherapy [22]. GBM microenvironment contains various immune cell categories, such as regulatory T cells (Tregs), tumor-associated macrophages (TAM), microglia, and suppressor cells from bone marrow [23]. Evidence has indicated that the expression of proinflammatory cytokines (IL-12, IL-18, and TNF-*γ*) was reduced, while soluble inhibitory molecules (IL-10 and VEGF) were enhanced in GBM [24, 25]. Glioma cells could also inhibit the antitumor immune response by regulating the activity of immune cells [26]. This study examined the significant variances in the immune microenvironment of three subtypes. We observed an increased percentage of neutrophils in iC2 compared to other subtypes. In the end, the three subtypes exhibited distinct immune microenvironmental characteristics. This change might be associated with their heterologous clinical consequences and therefore was prospective marks for BMG immunotherapy.

In addition, through contrasting the molecular characters, three illustrative markers (OSMR, IGFBP6, and MYBPH) were recognized and confirmed in the three subtypes. Myosin binding protein H (MYBPH) comprises 477 amino acids, and its molecular weight is 55 kDa [27]. The myosin-binding protein family contains two subtypes of MYBPH and MYBPC, which have apparent homology at the carboxyl end and have the same sequence and structural similarity [28]. Emerging evidence indicates that elevated MYBPH has been associated with a poor prognosis and recurrent in GBM [29]. Moreover, the deletion of MYBPH could inhibit the migration of glioma cells [30].

IGFBP is a group of multifunctional proteins with similar structure and function, and it has a high affinity with IGFs. IGFBP is vital in regulating physiological and pathological processes in vivo through IGF-dependent or IGF-independent mechanisms [31]. IGFBP-6 is a critical member of the IGF family and widely exists in human tissues, cells, and body fluids; it can bind to IGF-2 and inhibit the physiological function of promoting cell growth, proliferation, and differentiation mediated by IGF-2 [32]. IGFBP-6 could promote cell migration and regulate neutrophil activity, which suggests regulating inflammatory immune response and oxidative stress [33, 34]. Some studies have indicated that IGFBP-6 could inhibit tumor angiogenesis in multiple systems through the IGF-2-independent pathway [35].

The Oncostatin M receptor (OSMR) is a member of the interleukin-6 receptor family, performing various cellular functions, including regulating homeostasis, cell growth, and differentiation [36]. OSMR binds with gp130 to form a high-affinity receptor for its main ligand cytokine, antitumor M (OSM). OSM is mainly secreted by T lymphocytes, neutrophils, and macrophages and was initially used as an anticancer drug [37]. However, in some cases, OSM can promote tumor progression. Overexpression of OSM and OSMR has been detected in various cancers, including gastric, colorectal, breast, and glioma [38, 39]. OSM-OSMR signal transduction plays a vital role in inflammation, oxidative stress, hematopoiesis, and development and is increasingly considered an essential factor in tumor progression [40].

We observed that MYBPH and IGFBP6 were markedly connected to GBM diagnosis among the three genes. MYBPH and IGFBP6 were increased in iC3 and negatively connected to MET and prospective marks for BMG diagnosis.

In conclusion, we investigated underlying mechanisms of glioblastoma multiforme by multiomics exploration for genomics, epigenomics, and transcriptomics. We revealed that DNA CNV and MET change function critical roles in GBM. Moreover, we recognized three molecular subtypes of GBM and found three oxidative stress-related biomarkers. These findings might sustain the progression of exact diagnostic evaluations and therapies for GBM patients.

## Figures and Tables

**Figure 1:** Correlation analysis for MET-Gs and CNV-Gs. (a) Correlation analysis between MET-Gs and CNV-Gs in a *z*-score distribution. (b) CNV-G and MET-G overlap. (c) Distribution of CNV-Gs on chromosomes. (d) Distribution of MET-Gs on chromosomes. (e) The proportional frequency of CpG sites in the promoter based on the existence of CpG island. (f) The proportional frequency of CpG sites in the promoter is based on their distance from genomic regions.

**Figure 2:** CNV-Gs and MET-Gs gene set-based molecular subtype detection. (a) NMF clustering consequences for CNV-Gs. (b) NMF clustering consequences for MET-Gs. (c) The survival analysis for CNV-G subclasses. (d) The survival analysis for MET-G subclasses. (e) The overlapped subtypes recognized from CNV-G and MET-G clusters.

**Figure 3:** Integrated cluster sampling of CNV, EXP, and MET. (a) Heatmap of the expression of subtypes CNV-Gs and MET-Gs. (b) The difference of OS time between the three subtypes. (c) The difference of OS time between iC1 and iC2 subtypes. (d) The difference of OS time between iC1 and iC3 subtypes. (e) The difference of OS time between iC2 and iC3 subtypes.

**Figure 4:** DNA CNV abnormalities were accordant with MET abnormalities. (a) Frequency scattering of gain and loss in CNV. (b) Frequency scattering of gain and MetHyper in CNV. (c) CNV gain and MetHypo distribution (d) CNV loss and MetHyper distribution and MetHypo. (e) CNV loss and MetHypo distribution. (f) Frequency scattering of MetHyper and MetHypo.

**Figure 5:** Analysis of tumor immune cell infiltration in molecular subtypes. (a) Comparison of tumor immune cell infiltration in molecular subtypes. (b) The proportion of infiltrating immune cells in tissue samples. (c) Immunosignature scores of immune cells in molecular subtypes.

**Figure 6:** Subtype characterizations. (a) Distribution of CNV in the three subtypes. (b) Distribution of MET in the three subtypes. (c) Heatmap of DEGs in the three subtypes. (d) GO enrichment analysis for DEGs in three subtypes. (e) KEGG enrichment analysis for DEGs in three subtypes.

**Figure 7:** Association between gene expressions and CNV/MET. (a) Correlation between MYBPH CNV and expression in subtypes. (b) Correlation between IGFBP6 CNV and expression in subtypes; methylation and expression of the MYBPH gene. (c) Correlation between MYBPH MET and expression in subtypes. (d) Correlation between IGFBP6 MET and expression in subtypes. (e) The expression distribution of MYBPH in subtypes. (f) The expression distribution of IGFBP6 in subtypes. (g) The overall survival was examined for MYBPH. (h) The overall survival was examined for IGFBP6.

**Figure 8:** Mutation spectrum of the three GMB subtypes. (a–c) The top 50 mutated genes in the iC1, iC2, and iC3 subtypes. (d) Number of mutations in the top 50 genes. (e) Mutation spectrum of the first ten genes in the iC2 subtype.

## Data Availability

The labeled dataset used to support the findings of this study is available from the corresponding author upon request.
